# Morpho-physiological and biochemical attributes of Chili (*Capsicum annum* L.) genotypes grown under varying salinity levels

This article has been retracted.

**DOI:** 10.1371/journal.pone.0257893

**Published:** 2021-11-04

**Authors:** Madiha Butt, Abdul Sattar, Tahira Abbas, Rashid Hussain, Muhammad Ijaz, Ahmad Sher, Umbreen Shahzad, Sami Ullah, Marian Brestic, Marek Zivcak, Kristina Gasparovic, Bandar S. Aljuaid, Ahmed M. El-Shehawi, Ali Tan Kee Zuan

**Affiliations:** 1 College of Agriculture, Bahauddin Zakariya University, Bahadur Sub-Campus Layyah, Layyah, Pakistan; 2 Department of Horticultural Sciences, University College of Agriculture and Environmental Sciences, The Islamia University of Bahawalpur, Bahawalpur, Pakistan; 3 Department of Horticulture, MNS- Agriculture University, Multan, Pakistan; 4 Department of Plant Physiology, Slovak University of Agriculture, Nitra, Slovakia; 5 Department of Botany and Plant Physiology, Faculty of Agrobiology, Food, and Natural Resources, Czech University of Life Sciences Prague, Prague, Czech Republic; 6 Department of Biotechnology, College of Science, Taif University, Taif, Saudi Arabia; 7 Department of Land Management, Faculty of Agriculture, Universiti Putra Malaysia, Serdang, Selangor, Malaysia; Harran Üniversitesi: Harran Universitesi, TURKEY

## Abstract

Climate change is causing soil salinization, resulting in huge crop losses throughout the world. Multiple physiological and biochemical pathways determine the ability of plants to tolerate salt stress. Chili (*Capsicum annum* L.) is a salt-susceptible crop; therefore, its growth and yield is negatively impacted by salinity. Irreversible damage at cell level and photo inhibition due to high production of reactive oxygen species (ROS) and less CO_2_ availability caused by water stress is directly linked with salinity. A pot experiment was conducted to determine the impact of five NaCl salinity levels, i.e., 0,1.5, 3.0, 5.0 and 7.0 dS m^-1^ on growth, biochemical attributes and yield of two chili genotypes (‘Plahi’ and ‘A-120’). Salinity stress significantly reduced fresh and dry weight, relative water contents, water use efficiency, leaf osmotic potential, glycine betaine (GB) contents, photosynthetic rate (A), transpiration rate (E), stomatal conductance (Ci), and chlorophyll contents of tested genotypes. Salinity stress significantly enhanced malondialdehyde (MDA) contents and activities of the enzymatic antioxidants such as superoxide dismutase (SOD), catalase (CAT) and peroxidase (POD). In addition, increasing salinity levels significantly reduced the tissue phosphorus and potassium concentrations, while enhanced the tissue sodium and chloride concentrations. Genotype ‘Plahi’ had better growth and biochemical attributes compared to ‘A-120’. Therefore, ‘Plahi’ is recommended for saline areas to improve chili production.

## Introduction

Soil salinization is increasing day by day due to low rainfall, high evapotranspiration, poor soil and water management practices, which is affecting land fertility and resulting in poor productivity [1, 2]. It is estimated that salinity disrupts 19.5% of irrigated land and 2.1% dry land agriculture globally. In arid and semi-arid regions, salinity affects 25% irrigated lands [3], whereas in Pakistan, approximately 6.3 Mha of land is salt affected [4, 5]. One of the current challenges throughout the world is to promote food production for meeting increasing food demands. Global food production should increase by 38% till 2025 and by 57% until 2050 from current levels [6]. Increased sodium (Na^+^) concentration in plants constrains the growth and development of important horticultural crops through osmotic, ionic and oxidative stresses [7, 8].

Understanding the response of chili and mechanisms of resistance to salinity stress may help to contrive various approaches for improved performance under salt-affected conditions. Salt-affected plants wilt due to increased accumulation of soluble salts [Na^+^ and chloride (Cl^-^)], which disturb the normal growth and productivity of many essential crops, including vegetables [9]. Different plants have acquired different mechanisms to cope with salinity. Leaf stomatal conductance regulates the water evaporation losses to decrease osmotic stress under salinity. However, CO_2_ flux is inhibited due to the closure of stomata, and ultimately photosynthesis is negatively affected [10, 11].

Osmotic stress in plants is often associated with ion accumulation that causes nutritional imbalance and specific ion effects mainly due to Na^+^ and Cl^-^ toxicity, which hinders the uptake of essential nutrients such as potassium (K) and calcium (Ca) [12–15]. Due to nutritional imbalance, K^+^/Na^+^ ratio tend to decrease under salinity stress as excessive Na^+^ replaces K^+^ ions in plant tissue or enhance leakage of K^+^ from the cell by stimulating K^+^ efflux channels [16]. Meanwhile, reactive oxygen species (ROS) produced in plant cells due to salinity often damage biological membranes, proteins and nucleic acids [17]. An efficient system of enzymatic antioxidants, i.e., superoxide dismutase (SOD), peroxidase (POX) and catalase (CAT) are involved to detoxify these ROS [18, 19]. Different plant species such as tomato (*Solanum lycopersicum* (L.) H. Karst.), pea (*Pisum sativum* L.), chili (*Capsicum annum* L.), beans (*Phaseolus vulgaris* L.), jatropha (*Jatropha curcas* L.) and *Calendula* exhibit an upregulated activity of antioxidants under increased salinity [20, 21].

The ongoing problem of salinity has seriously hampered growth and yield of nutritionally important crops such as chilies. Chili despite being sensitive to salinity, is a good source of natural colors and antioxidant compounds that are essential for human health [22, 23]. Salinity substantially decreases the chlorophyll contents and enhances the proline contents and antioxidant activity in chili [24], which severely hampers its growth and yield [25]. Since chili is considered one of the most sensitive crops to salinity, we hypothesized that imposition of salinity to greenhouse-grown, potted plants of different chili genotypes would allow the analysis of the mechanisms of biochemical and physiological adaptation. The major objective of the study was to infer the salinity tolerance of different chili genotypes and morpho-physiological mechanisms involved in the tolerance to imposed salinity.

## Materials and methods

### Plant materials and growth conditions

The experiment was done in the greenhouse of the Institute of Horticultural Sciences, University of Agriculture, Faisalabad to evaluate the effect of salt stress on morphological, physiological, ionic and antioxidant activity of two chili genotypes, i.e., ‘Plahi’ and ‘A-120’. The study was exempt from permits as it did not involve any endangered species. Pre-soaked seeds of chili genotypes in sodium hypochlorite (30%) for 15 minutes were washed 2–3 times with deionized water [26] before sowing in 9L plastic pots filled with 8 kg sand. The pots were irrigated with Hoagland nutrient solution in two-day intervals. The temperature ranged between 25 and 30°C in greenhouse. Salinity treatments (i.e., 0, 15, 30, 50 and 70 mM NaCl) were initiated fifteen days after germination. Salinity was imposed in two equal splits with two-day interval. The plants were harvested after one week of second salinity split to determine morphological, gaseous exchange, ionic and biochemical attributes.

### Measurement of growth attributes

Shoot and root lengths (cm), and plant fresh and dry biomass (g) were measured after rinsing plant samples with deionized water. The samples were dried at 80°C for 48 hours to record dry biomass.

The dried samples were ground to fine powder for the determination of Na^+^ and K^+^ as described by Wolf [27]. For Cl^-^ contents, 1g sample was taken in 20 mL tubes filled with distilled water (20 mL) and heated overnight at 65°C. The extract was collected after filtration with filter paper to determine Cl^-^ contents using chloride analyzer (Corning-920, Germany).

Relative water contents (RWC) were measured from fully expanded uniform leaves by the method given by Sairam et al. [28]. Fresh weight of samples was recorded and then dipped in deionized water for 24 hours. The dipped samples were weighed to record turgid weight and then oven dried at 80°C for 48 hours to record dry weight. Relative water contents were determined according to Eq 1.


$$RWC\;(\%)=\frac{FW-DW}{TW-DW}\times 100$$ Eq 1

Here, FW = fresh weight (g), DW = dry weight (g) and TW = turgid weight (g) of leaf samples.

Leaf water potential was recorded from fully expanded leaves using gasket of the pressure chamber (Model, 615, USA). The same leaf sample was stored at -20°C for one week and then used to record osmotic potential (Vapro-5520, Wescor Inc. U.S.A).

### Measurement of gas exchange parameters and chlorophyll contents

Infrared gas analyzer (IRGA) (Analytical Development Company, Hoddesdon, England) was used for the determination of gas exchange traits like photosynthetic rate, transpiration rate and stomatal conductance [29]. Water use efficiency (WUE) was determined as a ratio of photosynthetic rate (A) and transpiration rate (E).

### Measurement of osmolytes

The method described by Heath and Packer [30] for the estimation of malondialdehyde contents (MDA) was opted. The reaction mixture contained leaf extract, 0.5% (w/v) Tri Butyric acid (TBA) solution and 20% (W/V) trichloroacetic acid (TCA) in equal concentration, whereas MDA was estimated at 532 and 600 nm wavelength [31]. A 0.5 g fresh leaf tissue was homogenized in 10 mL, 3% sulfosalicylic acid solution was added, and absorbance was recorded at 520 nm by double beam spectrophotometer (Hitachi-120, Japan).

### Measurement of the activities of antioxidant enzymes

The activities of antioxidant enzymes, i.e., SOD, CAT and POD were determined following the methods of Giannopolitis and Ries [32] and Chance and Maehly [33], respectively. The activity of each enzyme was expressed based on protein content.

### Statistical analysis

The experiment was laid out according to randomized complete block design with factorial arrangements. Chili genotypes were main factor, whereas salinity levels were regarded as sub-factors. Two-way analysis of variance (ANOVA) procedure in general linear models was used to test the significance in the data. Means were compared by Turkey’s honestly significant difference post-hoc test at 5% probability where ANOVA indicated significant differences. All statistical computations were done on Statistix 8.1 (Analytical Software 2005) software. Each treatment consisted of four replications and each replicate contained 3 plants of each genotype. The graphical presentation of data was done by using Sigma Plot.

## Results and discussion

### Growth parameters

Salt stress significantly altered growth of both chili genotypes. Among tested genotypes, ‘Plahi’ exhibited improved salt tolerance by producing 38% more fresh weight (1.13 g) than 0.70 g recorded in ‘A-120’ at 70 mM salinity (Fig 1). Similar observations were recorded for dry weight under control and saline environments. Under non-saline conditions, dry weight of ‘Plahi’ was 0.31g compared with 0.28 g recorded for ‘A-120’. Dry weight of both genotypes was decreased with increasing NaCl concentrations and minimum dry weight was recorded under 70 mM salinity with 0.15 g observed for ‘Plahi’ and 0.09 g for ‘A-120’.

**Fig 1:** Effect of NaCl stress on plant biomass of two chili genotypes.

Growth attributes (in root fresh weight, root dry weight, shoot fresh weight, and shoot dry weight) of genotype ‘Plahi’ were less affected by imposed salinity compared to genotype ‘A-120’. The negative effects on growth attributes of chili genotypes might be attributed to ionic imbalance and lower metabolic activities due to imposed salinity. Low water availability, osmotic stress and deficiency of minerals due to high salt concentration in rhizosphere could be an explanation for reduced growth attributes. Cell division and rate of cell expansion also decline with increased salinity, which reduce plant biomass [34]. Reduction in growth rates of salt-affected chili genotypes agrees with previous findings reported in various studies [35–37].

### Water relations

Relative water contents (RWC) and water use efficiency (WUE) showed a differential response in both chili genotypes and were considerably decreased with the increasing salinity (Fig 2). Chili plants under non-saline conditions (0 mM NaCl) expressed the highest RWC with 87.5% in ‘A-120’ and 86% in ‘Plahi’ genotypes. However, RWC significantly declined under increasing the salt concentrations and the lowest value (43%) was noted for ‘Plahi’ and ‘A-120’ (25%) genotypes under 70 mM salt stress. In the meantime, WUE of both genotypes decreased under saline conditions and the lowest values were recorded under 70 mM salt stress followed by 50 mM, 30 mM and 15 mM.

**Fig 2:** Effect of NaCl stress on relative water content and water use efficiency of two chili genotypes.

The RWC express water status of plant, which decreased with increase in salinity level. However, this decrease was more pronounced in ‘A-120’ genotype. Osmotic stress caused by salinity modifies water status of the plant in terms of water and osmotic potential. Water and osmotic potentials were significantly reduced in both genotypes. The toxic ions level was lower in ‘Plahi’ genotype, which might be attributed to less modification in water potential under stressed conditions and maintained higher turgor potential. The results are in conformity with several earlier studies [38–42].

### Effect of salinity on glycine betaine (GB) and malondialdehyde contents (MDA)

Glycine betaine contents of both genotypes showed an increasing tendency from lower to higher salinity concentrations to overcome salinity stress. Genotype ‘Plahi’ exhibited 22.4% higher glycine betaine contents over genotype ‘A-120’ under control conditions, whereas ‘Plahi’ exhibited 22% higher mean values of glycine betaine subjected to 70 mM salinity (Fig 3). Likewise, ‘Plahi’ contained 2.9 μmol g^-1^ f. wt. proline contents compared to 2.75 μmol g^-1^ f. wt. in ‘A-120’ under non-saline conditions. Likewise, ‘Plahi’ plants at 70 mM salt stress exhibited 17.15% more proline contents than ‘A-120’. However, MDA contents increased with increasing salinity and maximum MDA values for both genotypes were noted under 70 mM salinity. Genotype ‘A-120’ exhibited higher MDA contents (15.3 μmol kg^-1^ FW) than ‘Plahi’ genotype exposed to 70 mM salinity. Genotype ‘A-120’ surpassed ‘Plahi’ in terms of MDA contents, which shows its higher susceptibility to salt stress. The ability to maintain low levels of MDA conferred salt tolerance to ‘Plahi’ genotype which is in accordance with Liang et al. [43] and Ruiz et al. [44] in other crops.

**Fig 3:** Effect of NaCl stress on glycine betaine and MDA content of two chili genotypes.

Compatible solutes offer osmotic adjustment and sustain the macromolecular activity, most probably via ROS scavenging [45]. It is an important protective mechanism to cope with various stresses [46]. Salt-tolerant plants have higher proline accumulation capability [47]. It is noticed at vegetative growth phase of the plant as compared to reproductive phase [48]. Proline accumulation was also noticed by Miranda et al. [49], which supports the finding of current study.

Glycine betaine (GB) is significantly attributed to cell osmotic adjustment under stress conditions. It has protective role in maintaining leaf anatomy against salt stress [50]. The genotype ‘Plahi’ accumulated higher amount of GB than ‘A-120’ genotype; consequently, became more efficient in undoing harmful impacts of salinity. Higher accumulation of compatible solutes in ‘Plahi’ genotype its higher salt tolerance potential. These findings are also supported by Hajlaoui et al. [51] and Hassine and Lutts [52].

### Gas exchange attributes and chlorophyll contents

As expected, salinity had a significant impact on the photosynthetic rate of both genotypes and the highest photosynthesis rate was recorded under non-saline conditions (Figs 4 and 5).

**Fig 4:** Effect of NaCl stress on photosynthetic rate (A) and transpiration rate (B) of two chili genotypes.

**Fig 5:** Effect of NaCl Salt stress on stomatal conductance (Ci) and chlorophyll contents (SPA value) of two chili genotype.

Photosynthesis rate differed variably among genotypes grown under normal and saline environment. Genotype ‘Plahi’ observed higher photosynthesis rate even under increasing salinity. Genotype ‘Plahi’ showed improved characteristics and maintained about 61.5% higher photosynthesis rate than ‘A-120’ even under 70 mM salinity. Significantly higher transpiration rate was recorded for the plants grown under non-saline environments than the plants exposed to salinity. The highest transpiration rate was recorded for ‘Plahi’ genotype under saline and non-saline conditions. All salinity concentrations reduced transpiration rate of both genotypes; however, transpiration rate in ‘Plahi’ genotype was 51.2% higher than ‘A-120’ genotype under 70 mM salinity. Likewise, stomatal conductance was decreased under salt stress. Constant decline in stomatal conductance was recorded with increasing salinity and the highest decline was noticed under 70 mM salinity in both genotypes. However, ‘Plahi’ genotype had improved stomatal conductance under all salinity levels than genotype ‘A-120’.

Chlorophyll contents of both genotypes were significantly higher under non-saline growing conditions and reduced with imposed salinity. However, higher loss in chlorophyll contents recorded under increased salinity level. Besides, ‘Plahi’ genotype maintained higher chlorophyll contents than ‘A-120’ genotype. Reduction in chlorophyll contents was more pronounced in ‘A-120’ (33.3%) under 70 mM salinity than ‘Plahi’ genotype.

Photosynthetic apparatus is drastically impacted by salt stress [13]. It is evidenced with the negative impacts on CO_2_ assimilation rate, transpiration rate, stomatal conductance and water use efficiency (WUE) in both chili genotypes. Ionic imbalance created by salt stress might be responsible for altered physiological mechanisms. Similarly, stomatal movement irregularities and consequently less CO_2_ concentration stimulate photochemical damages. Imbalance of ions, especially for potassium and poor water status of salt-affected plants impair stomatal movements, which further lead to reduced photosynthesis and transpiration rates [53]. Photosynthesis rate also declines due to photosystem damages under low CO_2_ availability. Broadly, declined photosynthesis rate under salt stress is due to low CO_2_ availability [54], changes in photosynthetic metabolism [55], photochemical apparatus modifications [56] and stomatal closure [57–59]. Higher tolerance of ‘Plahi’ genotype to salinity is the result of higher potassium concentration in its leaf tissues, which resultantly supported stomatal movements and maintained physiological mechanisms. This property of ‘Plahi’ genotype also suggested for higher WUE, which describes maximum utilization of plant resources in producing plant biomass, as evidenced by Ali et al. [53] and Ashraf [60].

### Effect of salinity on antioxidative enzyme activities

Results revealed increased antioxidant enzymes’ activities in chili plants subjected to different salinity concentrations (Fig 6). Chili plant grown under non-saline conditions recorded reduced enzymatic activities compared to the plants grown under salt stress. The activities of SOD, CAT and POD were dependent on salinity concentration and maximum activities were observed under 70 mM salinity level. Genotype ‘Plahi’ proved superior over ‘A-120’ by exhibiting 28%, 27% and 48% higher activities of SOD, CAT and POD enzymes under 70 mM salinity.

**Fig 6:** Effect of NaCl stress on antioxidant enzymatic activities (SOD, CAT & POD) of two chili genotypes.

The tested genotypes in the current study responded to salt stress by exhibiting higher activities of SOD, POD and CAT. The enzyme activity was more pronounced in ‘Plahi’ than ‘A-120’ genotype, which evidenced its higher salt-tolerance through detoxifying ROS. These findings are supported by Heidari [61], Sergio et al. [62] and Miranda et al. [49].

### Effect of salinity on sodium and potassium contents

Sodium (Na^+^) and K^+^ contents of the plants exposed to salinity stress increased significantly compared to plants grown under non-saline conditions (Fig 7). Genotype ‘Plahi’ observed reduced accumulation of Na^+^ and Cl^-^ contents under all salinity levels. Genotype ‘Plahi’ exhibited significantly reduced Na^+^ under 70 mM salinity (Figure). On the other hand, higher K^+^ ions were recorded in both genotypes under non-saline conditions. Results indicated that K^+^ contents declined with increasing salinity levels; however, a decline of K^+^ contents was more prominent in ‘A-120’ genotype. The increase in dissolved solutes and ions under salt stress and reduced water availability contributed towards reduced water and osmotic potential of plants [38, 51, 59]. Salt-tolerance of the plants can be attributed to their ability of reduced absorption and transport of toxic ion like Na^+^ and Cl^-^ to above ground strata. Since salinity hinders the absorption of beneficial ions like calcium and potassium, so the plant with capability to show more absorption of these ions will have higher salt tolerance potential.

**Fig 7:** Effect of NaCl stress on ionic contents (sodium & potassium) of two chili genotypes.

## Conclusion

In conclusion, current study suggests that ‘Plahi’ genotype has better salt-tolerance because of higher relative water contents, water use efficiency, leaf osmotic potential, glycine betaine (GB) contents, photosynthetic rate (A), transpiration rate (E) and stomatal conductance (Ci) under salt stress. In addition, higher activities of the enzymatic antioxidants such as superoxide dismutase (SOD), catalase (CAT) and peroxidase (POD) can provide faster recovery from salt damage in salt-tolerant chili genotypes. Hence, ‘Plahi’ genotype is recommended for saline areas to improve chili production.
